The article "Interferon and Ribavirin Combination Treatment Synergistically Inhibit HCV Internal Ribosome Entry Site Mediated Translation at the Level of Polyribosome Formation" was retracted in 2024. Reasons: duplicated images; overlap with earlier publications; original data or images not available; unreliable results or conclusions.

# Interferon and Ribavirin Combination Treatment Synergistically Inhibit HCV Internal Ribosome Entry Site Mediated Translation at the Level of Polyribosome Formation

**DOI:** 10.1371/journal.pone.0072791

**Published:** 2013-08-23

**Authors:** Rajesh Panigrahi, Sidhartha Hazari, Sruti Chandra, Partha K. Chandra, Sibnarayan Datta, Ramazan Kurt, Craig E. Cameron, Zhuhui Huang, Haitao Zhang, Robert F. Garry, Luis A. Balart, Srikanta Dash

**Affiliations:** 1 Pathology and Laboratory Medicine, Tulane University School of Medicine, New Orleans, Louisiana, United States of America; 2 Micribiology and Immunology, Tulane University School of Medicine, New Orleans, Louisiana, United States of America; 3 Gastroenterology, Hepatology and Medicine, Tulane University School of Medicine, New Orleans, Louisiana, United States of America; 4 Department of Biochemistry and Molecular Biology, Penn State University, University Park, United States of America; 5 Hepatitis Research Program, Southern Research Institute, Frederick, Maryland, United States of America; Saint Louis University, United States of America

## Abstract

**Purpose:**

Although chronic hepatitis C virus (HCV) infection has been treated with the combination of interferon alpha (IFN-α) and ribavirin (RBV) for over a decade, the mechanism of antiviral synergy is not well understood. We aimed to determine the synergistic antiviral mechanisms of IFN-α and RBV combination treatment using HCV cell culture.

**Methods:**

The antiviral efficacy of IFN-α, RBV alone and in combination was quantitatively measured using HCV infected and replicon cell culture. Direct antiviral activity of these two drugs at the level of HCV internal ribosome entry site (IRES) mediated translation in Huh-7 cell culture was investigated. The synergistic antiviral effect of IFN-α and RBV combination treatment was verified using both the CalcuSyn Software and MacSynergy Software.

**Results:**

RBV combination with IFN-α efficiently inhibits HCV replication cell culture. Our results demonstrate that IFN-α, interferon lambda (IFN-λ) and RBV each inhibit the expression of HCV IRES-GFP and that they have a minimal effect on the expression of GFP in which the translation is not IRES dependent. The combination treatments of RBV along with IFN-α or IFN-λ were highly synergistic with combination indexes <1. We show that IFN-α treatment induce levels of PKR and eIF2α phosphorylation that prevented ribosome loading of the HCV IRES-GFP mRNA. Silencing of PKR expression in Huh-7 cells prevented the inhibitory effect of IFN-α on HCV IRES-GFP expression. RBV also blocked polyribosome loading of HCV-IRES mRNA through the inhibition of cellular IMPDH activity, and induced PKR and eIF2α phosphorylation. Knockdown of PKR or IMPDH prevented RBV induced HCV IRES-GFP translation.

The article "Interferon and Ribavirin Combination Treatment Synergistically Inhibit HCV Internal Ribosome Entry Site Mediated Translation at the Level of Polyribosome Formation" was retracted in 2024. Reasons: duplicated images; overlap with earlier publications; original data or images not available; unreliable results or conclusions.

**Conclusions:**

We demonstrated both IFN-α and RBV inhibit HCV IRES through prevention of polyribosome formation. The combination of IFN-α and RBV treatment synergistically inhibits HCV IRES translation via using two different mechanisms involving PKR activation and depletion of intracellular guanosine pool through inhibition of IMPDH.

## Introduction

HCV infection leads to a fast progression to chronic liver disease, liver cirrhosis and hepatocellular carcinoma [1]. There are 160 million people infected with HCV representing a major public health problem worldwide [2]. HCV is an enveloped positive-stranded RNA virus that belongs to the *Flaviviridae* family. This family includes yellow fever and dengue viruses, which also affect humans [3]. The genome of HCV is organized into a highly conserved 5’-untranslated region (5’ UTR), a large open reading frame (ORF) and a 3’-untranslated region (3’ UTR). The 5’ UTR of HCV genome binds to the host ribosome using the internal ribosome entry site (IRES) mechanism that facilitates translation of HCV protein [3,4]. The HCV genome contains a large open reading frame (ORF) that encodes for a polyprotein 3011 amino acid long. The polyprotein is proteolytically processed in the endoplasmic reticulum (ER) membrane into 10 different mature viral proteins by the cellular and viral protease [3]. The core protein and the two glycoproteins E1 and E2 are structural proteins; they are required for the formation of the viral particle, as well as assembly, export and infection. The non-structural (NS) proteins include the p7 ion channel, the NS2 protease, the NS3 serine protease and RNA helicase, the NS4A polypeptide (a cofactor for NS3 protease), the NS4B, the NS5A protein, and the NS5B RNA-dependent RNA polymerase, which are required for replication of the viral genome. The NS proteins (protease and polymerase) have been the targets of intense research efforts for the development of antiviral drugs against HCV. The highly conserved 3’ UTR present at the very end of the HCV genome is important for the initiation of viral RNA replication [5]. HCV infection is initiated by the attachment and entry of virus particles into the host cells by receptor mediated endocytosis [6].

IFN-α and RBV, along with one of the protease inhibitors, is the standard-of-care for chronic HCV 1a infection [7]. Recently the FDA approved two protease inhibitors (Telaprevir and Boceprevir) that are specific to HCV genotype 1 virus NS3 sequences. IFN-α in combination with RBV is still used as the standard treatment for other HCV genotypes. Ribavirin is a guanosine analogue used for the treatment of a number of RNA viruses including the respiratory syncytial virus (RSV), Lass fever virus and HCV [8]. IFN-α and RBV combination therapy is more effective in the treatment of chronic HCV infection than treatment with a single agent [9]. Ribavirin is a synthtic guanosine nucleoside analogue (1-b-D-ribofuranosyl-1,2,4-triazole-3-carboxamide) which has been shown to be metabolized intracellularly into ribavirin mono (RMP), di- (RDP) and triphosphate (RTP) [10]. Although RBV is extensively used to treat patients with HCV-infection the direct antiviral mechanism by which the compound inhibits viral replication remains largely elusive [8]. Furthermore, the mechanism by which the combination of RBV and IFN-α combination improves the treatment response is unclear [11]. Understanding the synergistic antiviral mechanisms of IFN-α and RBV action using the improved HCV cell culture system is important and may open new therapeutic interventions to improve the clinical response.

The article "Interferon and Ribavirin Combination Treatment Synergistically Inhibit HCV Internal Ribosome Entry Site Mediated Translation at the Level of Polyribosome Formation" was retracted in 2024. Reasons: duplicated images; overlap with earlier publications; original data or images not available; unreliable results or conclusions.

In our present study, we addressed the mechanism of IFN-α and RBV combination synergy by using full-length infectious cell culture, replicon model and a sub-genomic HCV IRES expression model. We observed that IFN-α and RBV each directly inhibited translation of HCV IRES by blocking polyribosome formation. Our results suggest that IFN-α and RBV each activate PKR and eIF-2α phosphorylation which blocks HCV IRES mediated translation and synergistically inhibits HCV replication. Furthermore, RBV mediated inhibition of IMPDH activity also contributes to the blockadge of polyribosome loading.

## Materials and Methods

### Cell culture and reagents

Human hepatoma cell lines, Huh-7 and Huh-7.5 were maintained in Dulbecco’s modified eagle’s medium (DMEM) supplemented with 10% fetal bovine serum (FBS), non-essential amino acids and sodium pyruvate. The stable S3-GFP replicon cell line (HCV JFH1 2a) was maintained in DMEM and 10% FBS supplemented with G-418 (1 µg/mL) as described in our previous study [12]. Full-length *Renilla* luciferase (Rluc) reporter based JFH-∆V3-Rluc clone used in our infectivity assay was a kind gift from Curt H. Hagedorn Laboratory [13]. A replication defective adenovirus that expresses T7 RNA polymerase (AdexCAT7) was a kind gift from Tatsuo Miyamura, National Institute of Infectious Disease, Tokyo, Japan [14]. Cell culture derived infectious HCV stocks were prepared from the supernatants of Huh-7.5 cells as described previously [15]. Recombinant IFN-α 2b (Intron-A) was purchased from Schering-Plough (New Jersey, USA). Ribavirin, Cycloheximide and Guanosine were purchased from Sigma Chemical Company (St. Louis, MO, USA). Interferon lambda 1 (IL-29) was obtained from Peprotech, Rocky Hills, NJ, USA.

The article "Interferon and Ribavirin Combination Treatment Synergistically Inhibit HCV Internal Ribosome Entry Site Mediated Translation at the Level of Polyribosome Formation" was retracted in 2024. Reasons: duplicated images; overlap with earlier publications; original data or images not available; unreliable results or conclusions.

### IFN-α and RBV combination treatment in sub-genomic replicon cell line and in infected HCV cell culture

S3-GFP replicon cells were cultured in presence of different concentrations of IFN-α and RBV alone and in combination for 72 hours. The antiviral effect of IFN-α and RBV combination treatment was evaluated by GFP expression under a fluorescence microscope and quantified by flow cytometric analysis. Huh-7.5 cells were infected with JFH-∆V3-Rluc virus (MOI 0.1) using a standard protocol [15]. After 48 hours, infected cultures were treated with increasing concentrations of IFN-α or RBV alone or in combination. After 72 hours, the antiviral effect of IFN-α and RBV treatment was measured by NS5A-Rluc activity. Total protein concentration was measured by the Bradford method and luciferase activity was expressed in per micro-gram of total protein. HCV core protein expression was also measured by immunocytochemistry using the following protocol. Infected Huh-7.5 cells with or without IFN-α treatment were mounted onto a glass slide via the cytospin method. The cells were washed in PBS, fixed in chilled acetone for 15 minutes and then permeabilized by Reveal Decloaker RTU (Biocare Medical, RV 100) reagent for 25 minutes. Slides were cooled for 25 minutes and blocking was performed with Background Sniper (Biocare Medical, BS966) for 10 minutes at room temperature. The cells were incubated with monoclonal anti-core antibody (Thermo Scientific, Pierce HCV-core antigen specific mouse monoclonal antibody, Ma1-080) at 1:200 diluted with Da Vinci Green Diluent (Biocare Medical, PD900) for 1 h at room temperature. Cells were washed three times in Tris-buffered saline (TBS) pH 8.0, and incubated with MACH 4 mouse probe (Biocare Medical, UP534) for 10 minutes and then incubated with MACH4 HRP Polymer (Biocare Medical, MRH534) for 30 minutes. Next, the cells were treated with diaminobenzidine (DAB) chromogen (Dako Cytomation, Carpinteria, CA) for 5 minutes. The slides were counterstained with hematoxylin for 30s and Tacha’s bluing Solution (Biocare Medical, HTBLU) for 30 s, dehydrated, mounted and observed by light microscopy.

### IFN-α and RBV effect on HCV-IRES mediated translation

A chimeric sub-genomic clone of HCV IRES and GFP (pHCV IRES-GFP) was used to determine the antiviral mechanisms of IFN-α and RBV as described previously [16]. Plasmids pEGFP-N1 and pDsRed-N1 expressing GFP and RFP (red fluorescence protein) respectively from a human cytomegalovirus (CMV) promoter by a non-IRES dependent mechanism were used as a control (BD Biosciences, Clonetech, Palo Alto, CA). Huh-7 cells (1X10^4^ cells/well) were infected with AdexCAT7 (10 pfu/cell) for 2 hours at 37^0^C, and then transfected with pHCVIRES-GFP clone using the X-tremeGENE 9 transfection reagent (Roche Diagnostics, Indianapolis, IN). The pEGFP-N1 and pDsRed-N1 plasmid was transfected without addition of AdexCAT7 to the cells. Huh-7 cells were first transfected with 1µg of HCV IRES-GFP or pEGFPN1 or pDsRedN1 plasmid and treated with IFN-α (10-1000 IU/mL) and RBV (10-40 µg/mL). After 24 hrs, GFP expression was monitored under a fluorescence microscope (Olympus IX 70, Germany) and quantified by flow cytometric analysis. Transfected cells were examined with a fluorescent microscope at 484 nm for the expression of GFP and at 340 nm for Hoechst 33342 stain. Nuclear stain was superimposed over cytoplasmic GFP using Adobe Photoshop computer software generated the images.

The article "Interferon and Ribavirin Combination Treatment Synergistically Inhibit HCV Internal Ribosome Entry Site Mediated Translation at the Level of Polyribosome Formation" was retracted in 2024. Reasons: duplicated images; overlap with earlier publications; original data or images not available; unreliable results or conclusions.

### Evaluation of synergy interaction at the level of HCV-IRES mediated translation

A Sub-genomic construct (pHCV-IRES-RLuc) with T7 promoter, HCV IRES-Rluc fusion, 3’ UTR of HCV, a cDNA copy of the autolytic ribozyme from antigenomic strand of the hepatitis delta virus and T7 transcriptional terminator sequences was used to study HCV-IRES mediated translation. Huh-7 cells were transfected with pHCV-IRES-RLuc plasmid using the same procedure described above. The cells were treated with IFN-α (10-1000 IU/mL) and RBV (10-80 µg/mL) alone and combination immediately after transfection and incubated at 37^o^C for 24 hours. After 24 hours, the cells were washed with PBS, lysed and *Renilla* luciferase activity was measured (Luman LB9507, EG & G, Berthold, Berlin, Germany). The consistency of the results was maintained by quantifying emissions from triplicate wells for each treatment. IFN-λ also shows good antiviral effect against HCV (unpublished data). To determine the combinatory effect of IFN-α, IFN-λ and RBV, Huh-7 cells transfected with pHCV-IRES-RLuc plasmid were treated with 0, 10, 100, 1000 IU/mL of IFN-α 0 10 20 50 100 μg/mL IFN-λ and 0, 10, 20, 40 µg/mL of RBV. *Renilla* luciferase values were analyzed by using the CalcuSyn software (Biosoft). This program uses the median-effect principle to delineate the interaction between these two drugs. For each combination, the program generates a combination index (CI) based on the equation below described by Chou et al [17,18]. A combination index (CI) of <1 means synergism, CI=1 means additive and CI>1 means antagonism. Drug–drug combination analysis of IFN-α and RBV was performed with the MacSynergy II program [19,20].

### Polyribosome fractionation and Northern blot analysis

To examine whether IFN-α and RBV treatment inhibits translation by preventing the loading of polyribosomes on the IRES-GFP mRNA, polysome analysis was performed using sucrose density gradient centrifugation. Huh-7 cells were transfected with pHCV IRES-GFP clone using a two-step transfection procedure. After transfection, cells were treated with IFN-α (1000 IU/mL) or RBV (40 µg/mL) and after 24 hours, the expression of GFP was examined. The polysome analysis was performed using a protocol described earlier [21]. Briefly, transfected Huh-7 cells were washed twice with ice-cold PBS pH-7.2 containing 100µg/mL cycloheximide. The cells were lysed by 200 µl of polysomes lysis buffer containing 100 mM KCl, 5mM MgCl_2_, 10 mM HEPES, pH7.4, 100 µg/mL cycloheximide, 0.5% Nonidet P-40, and 1000 units/mL RNase inhibitor (Ambion Inc, Austin, TX). The cell lysate was passed four times through a 27-gauge needle to ensure complete cell lysis. Nuclei were pelleted by centrifugation at 12,000 rpm for 5 minutes. The supernatant was collected and centrifuged an additional time to ensure the removal of any nuclei. The resulting supernatant was layered on a linear 15-60% (w/v) sucrose gradient in polysome gradient buffer (100 mM KCl, 5 mM Mg Cl_2_ and 10 mM HEPES pH 7.4) and centrifuged at 36,000 rpm for 2 hours at 4^°^C in a Beckman SW41 rotor. The distribution of ribosomal RNA along the sucrose density gradient fractions was determined using a polysome fractionator (Teledyne ISCO, Brandel, Inc, Gaithersburg, Maryland). Total RNA was isolated from the sucrose density fractions by treating with proteinase K solution (0.2 M Tris-HCl, pH 7.5, 25 mM EDTA, 0.3 M NaCl, 2% SDS, and 250 µg/mL proteinase K, RNase free DNase-I 10 U/mL). Half of the RNA samples were subjected to Northern blot analysis to examine the distribution of HCV IRES-GFP mRNA in each fraction. Identical experiments were performed to determine the effect of RBV on the distribution of HCV IRES-GFP mRNA in the polysome fractions. Control experiments were performed using the pEGFP-N1 plasmid to determine the effect of IFN-α on the distribution of mRNA in the polysome fraction whose translation occurs via cap-dependent mechanism. To detect the HCV-IRES mRNA in the polysome fractions an anti-sense ^32^P labeled riboprobe (10^6^ cpm/mL) targeted to the highly conserved 5’ UTR of HCV genome was used. To detect EGFP mRNA in the polysome fractions, an anti-sense ^32^P labeled RNA probe (10^6^ cpm/mL) targeted to the GFP was used. Northern hybridization was performed using the ULTRAhyb reagent (Ambion Inc, Austin, TX) at 68^0^C for 16 hours. Blots were then washed twice for 15 min each at 37^0^C using a washing solution (0.1X SSC-0.1% SDS), followed by two 15 min washes at 37^0^C using a washing solution (0.1X SSC-0.1% SDS). The membrane was exposed for autoradiography using Bio Max X-ray film (Kodak imaging system). Proteins bound to polyribosomes were isolated using a standard protocol [22]. Briefly, sucrose gradient fractions were precipitated by an addition of cold trichloroacetic acid to a final volume of 10% and were incubated on ice for 30 minutes. This step was followed by centrifugation at 20,000g for 15 min at 4°C. Pellets were washed once with 5% TCA and once with cold acetone. Finally, protein pellets were resuspended in a sample buffer (50 mM Tris at pH 6.8, 2% SDS, 2% glycerol) and 1% β-mercaptoethanol or 1 mM DTT, heated at 65°C, and processed for SDS-PAGE. Protein in the or transferred to nitrocellulose for Western blot.

The article "Interferon and Ribavirin Combination Treatment Synergistically Inhibit HCV Internal Ribosome Entry Site Mediated Translation at the Level of Polyribosome Formation" was retracted in 2024. Reasons: duplicated images; overlap with earlier publications; original data or images not available; unreliable results or conclusions.

### Western blot analysis

Protein lysates from cells were prepared after treatment with IFN-α and RBV for 24 hours. Equal amounts of protein were resolved on SDS-PAGE gels. The antibodies to PKR, eIF2α, peIF2α (Ser51), β-actin, PKR, anti-mouse IgG, and anti-rabbit IgG HRP-linked antibody were purchased from Cell Signaling, Beverly, MA. Antibody to p-PKR (pT446) was obtained from Epitomics, Burlingame, CA. Antibody to IMPDH was obtained from Santa Cruz, Dallas, USA. Twenty microgram of proteins were resuspended in sample buffer (50 mM Tris at pH 6.8, 2% SDS, 2% glycerol) and 1% β-mercaptoethanol or 1 mM DTT, heated at 65°C, and processed for SDS-PAGE. Proteins were transferred to nitrocellulose membrane and Western blotting was performed using a standard protocol.

### Knockdown of PKR and IMPDH mRNA

siRNA duplexes targeting the coding regions of human IMPDH1 (Qiagen, catalog no. SI02781044), PKR (Qiagen, SI02223018) and unrelated control siRNA were obtained from Qiagen. Huh7 cells were transfected with the indicated siRNA duplexes using Oligiofectamine (Invitrogen, CA). After 6 hours of siRNA treatment the cells were transfected with the IRES-GFP sub-genomic construct and then treated with either IFN-α or RBV to examine translational inhibition.

## Results

### IFN-α and RBV synergistically inhibit HCV replication in replicon and full-length infectious cell culture models

The genomic and sub-genomic clones for HCV genotype 2a used to develop the HCV replication model are shown (Figure **S1A**). We first measured the cytotoxic effects of IFN-α and RBV treatment alone and in various combinations using Huh-7 cells and S3-GFP replicon cell line by a MTT assay. Ribavirin up to 200 µg/mL did not show any cytotoxicity (Figure **S2A**). The viability of S3-GFP cells were more than 90% at 48 hours when treated with RBV (10-60 µg/mL) and IFN-α (10-1000 IU/mL) alone (Figure **S2B**) or in combination (Figure **S2C**). Based on the MTT assay results, concentration of RBV (10-40µg/ml) permitting high viability was used for subsequent antiviral assays. The antiviral effect of IFN-α and RBV combination treatment in S3-GFP replicon cells after 72 hours was confirmed by the measurement of GFP expression under a fluorescence microscope (Figure **1A**) and the expressed GFP was quantified by flow cytometric analysis (Figure **1B**). The sub-genomic replicon system does not produce infectious virus due to lack of the structural proteins. Antiviral effect of IFN-α and RBV combination treatment was measured using an infectious cell culture model using the JFH1-Rluc chimera virus. The IFN-α and RBV treatment gradually reduced the RLuc activity in a dose dependent manner (Figure **1C**). The inhibition of HCV replication was significant at RBV 20µg/mL with IFN-α (100 IU/mL) and RBV 40µg/mL with IFN-α (250 IU/mL). We verified the antiviral effect of combination treatment by measuring HCV core protein expression by immunostaining (Figure **1D**). The number of HCV core positive cells in five different high power fields (hpf) were counted and compared with untreated control (Figure **1E**).

The article "Interferon and Ribavirin Combination Treatment Synergistically Inhibit HCV Internal Ribosome Entry Site Mediated Translation at the Level of Polyribosome Formation" was retracted in 2024. Reasons: duplicated images; overlap with earlier publications; original data or images not available; unreliable results or conclusions.

**Figure 1:** Antiviral effect of IFN-α and RBV combination treatment using a sub-genomic replicon cell line (S3-GFP) and HCV infected Huh-7.5 cells. (**A**) S3-GFP cells were treated with IFN-α and RBV for 72 hours. GFP expression was examined under a fluorescence microscope. (**B**) GFP positive cells were quantified by flow cytometric analysis. (**C**) Infected Huh-7.5 cells were treated with IFN-α alone, RBV alone and combination for 72 hours. *Renilla* Luciferase activity of infected cells was measured and normalized with 1µg of cellular protein. (**D**) Expression of HCV core protein was measured by immunostaining and (**E**) core positive cells in five different high power fields (hpf) at 40X magnification were counted under a light microscope. Quantitative assessment of the number of HCV positive cells with mean and standard deviation of the combination treatment are compared.

### IFN-α, IFN-λ1 and RBV combination treatment synergistically inhibit HCV IRES mediated translation

Previously we reported that type I and Type II IFN inhibit HCV replication by targeting the 5’ UTR of HCV RNA genome used for IRES mediated translation [23]. Here we examined whether IFN-α and RBV combination treatment could also inhibit the HCV IRES mediated translation. The mechanisms of IFN-α and RBV action on HCV translation were examined using HCV IRES-GFP or HCV IRES-RLuc based subgenomic clones (Figure **S1B**). Plasmid clones pEGFP-N1 and pDsRed-N1 were used as controls to examine the effect of IFN-α and RBV treatment on the expression of GFP or RFP by non-IRES mechanisms (Figure **S1B**). High-level expression of GFP from HCV IRES in Huh-7 cells was achieved by using two-step transfection procedures that first involve infection with replication defective adenovirus that expresses T7 RNA polymerase (AdexCaT7), followed by transfection with a transcription plasmid (Figure **S1C**). The HCV IRES mediated translation of GFP was inhbited by both IFN-α and RBV at increasing concentration of both the drugs as evidenced by fluorescence imaging (Figure **2A**) and Western blot analysis (Figure **2B**). The cap dependent translation of GFP or RFP was not inhibited by addition of these two drugs (Figures **S3A** and **S3B**). IFN-α and RBV show maximum HCV IRES inhibition at 1000 IU/mL and 40 µg/mL respectively. Results of Northern blot analysis indicate that the intracellular IRES GFP mRNA is relatively stable in the IFN-α and RBV treatment. There is no significant difference in the stability of HCV IRES-GFP mRNA in Huh-7 cells treated with increasing concentrations of IFN-α (10 to 1000 IU/mL) compared to GAPDH mRNA level used as a control (data not shown). These results indicate that IFN-α and RBV treatment inhibit translation of HCV IRES-GFP without altering the stability of intracellular HCV IRES sub-genomic mRNA. Interferon lambda (IFN-λ1) is a type III IFN, which has been found to have a sustained antiviral activity against HCV (unpublished results). We quantified the relative antiviral activity of IFN-α, IFN-λ1 and RBV at the level of HCV IRES translation using a HCV IRES Rluc plasmid (Figure **S1B**). Huh-7 cells were transfected with HCVIRES-Rluc plasmid and then treated with different concentrations of IFN-α, IFN-λ1 and RBV alone and in combination. The antiviral activity of combination treatment was measured by *Renilla* luciferase activity per microgram of cellular protein. The results presented in Figure **3A** show that IFN-α, IFN-λ1 and RBV each inhibits HCV replication in a dose-dependent manner. The combination of IFN-α and IFN-λ1 at the level of HCV-IRESRLuc expression was examined (Figure **3B**). Combination treatment of IFN-α with RBV (Figure **3C**) and IFN-λ1 with RBV (Figure **3D**) showed a stronger inhibitory effect on HCV IRES-Rluc expression. Determination of a synergistic, additive or antagonstic effect of IFN-α and RBV combination was performed according to the median effect principle using the CalcuSyn computer program. The combination treatment of IFN-α and RBV was highly synergistic with CI values of <1. Results using CalcuSyn software revealed synergistic interactions across the entire range of RBV with either IFN-α or IFN-λ1 combinations tested (Figure **4A and 4B**). IFN-α and IFN-λ1 combination treatment did not show synergistic inhibition of the HCV IRES-translation (Figure **4C**). Analysis of IFN-α, IFN-λ1 and RBV treatment was subsequently performed with the MacSynergy II program. The MacSynergy II program calculated the theoretical additive interactions of the drugs based on the Bliss Independence mathematical definition of expected effects for drug–drug interactions. The additive interactions were calculated from the dose–response. If the interactions are additive, the resulting surface appeared as horizontal plane at 0% above the calculated additive surface in the resulting difference plot. Peaks above this plane is an indicative of synergy, while depression below the horizontal plane is an indication of antagonism. This analysis revealed that RBV treatment in combination with either IFN-α or IFN-λ1 had resulted in strong synergistic interactions (Figure **4G and 4H**). In contrast, IFN-α and IFN-λ1 combination treatment show slightly antagonistic interactions (Figure **4C and 4I**). Average cell inhibition was shown in Figure **4D, 4E** **and 4F**. In conclusion, synergistic interactions between RBV and IFN treatments were observed at physiologically relevant concentrations.

The article "Interferon and Ribavirin Combination Treatment Synergistically Inhibit HCV Internal Ribosome Entry Site Mediated Translation at the Level of Polyribosome Formation" was retracted in 2024. Reasons: duplicated images; overlap with earlier publications; original data or images not available; unreliable results or conclusions.

**Figure 2:** IFN-α and RBV each inhibited the internal ribosome entry site (IRES) mediated translation of green fluorescence protein (GFP). Huh-7 cells were infected with T7-expressing adenovirus. After 2 hrs, HCV IRES-GFP plasmid was transfected and then treated with indicated concentration of IFN-α and RBV. (**A**) HCV IRES mediated GFP expression was monitored under fluorescent microscopy. (**B**) Inhibition of GFP expression was further confirmed by Western blot analysis in both IRES and non-IRES mechanisms. β-actin is used as loading controls.

**Figure 3:** Different combinations of IFN-α, RBV, and IFN-λ inhibits HCV IRES Rluc mediated translation. Huh-7 cells were infected with T7-expressing adenovirus. After 2 hrs, HCV IRES-RLuc plasmid was transfected and then treated with indicated concentration of IFN-α, IFN-λ and RBV. The concentration dependent inhibition of *Renilla* luciferase activity by (**A**) IFN-α, RBV, and IFN-λ single treatment;(**B**) Combination of IFN-α + IFN-λ; (**C**) Combination of IFN-α + RBV and (**D**) Combination of IFN-λ + RBV.

**Figure 4:** Analysis for synergistic effect of IFN-α + IFN-λ, IFN-α + RBV, and IFN-λ + RBV using Calcusyn and MacSynergyII software. (**A**) CalcuSyn software analysis show that IFN-α + RBV combination treatment has a very strong synergy antiviral activity against HCV IRES mediated inhibition with combination index, CI<1. (**B**) IFN-λ + RBV combination treatment also has a very strong synergy antiviral activity with CI<1. (**C**) IFN-α + IFN-λ treatment are either additive or slightly antagonistic. Three dimensional inhibition plots of (**D**) IFN-α + RBV, (**E**) IFN-λ + RBV and (**F**) IFN-α + IFN-λ treatment against HCV IRES mediated inhibition of Rluc at 95% confidence interval synergy plot. Three dimensional synergy plot of (**G**) IFN-α + RBV, (**H**) IFN-λ + RBV, and (**I**) IFN-λ + IFN-α.

The article "Interferon and Ribavirin Combination Treatment Synergistically Inhibit HCV Internal Ribosome Entry Site Mediated Translation at the Level of Polyribosome Formation" was retracted in 2024. Reasons: duplicated images; overlap with earlier publications; original data or images not available; unreliable results or conclusions.

### IFN-α and RBV treatment prevents loading of polyribosome to HCV IRES containing mRNA

The translation of HCV genomic RNA is initiated by the binding of the host cell ribosome to a highly conserved RNA sequence called the internal ribosome entry site (IRES), located in the 5’ UTR. We examined whether inhibition of GFP expression in the HCV IRES subgenomic clone could have occurred due to a differential loading of polyribosome. The upper panel (Figure **5A**) shows the separation of 40S, 60S and 80S and polyribosme in the sucrose density gradient using a polysome fractionator (Teledyne ISCO, BRANDEL). Total RNA from each gradient fraction was isolated and analyzed by agarose gel electrophoresis. The location of monosomes and polysomes was determined by ethidium bromide staining (Figure **5B**). Polysome fractionation of IRES-GFP transfected Huh-7 cells after treatment with IFN-α or RBV was performed to examine distribution of HCV IRES-GFP mRNA in the monosome and polysome fractions. The amount of HCV IRES containing GFP mRNA associated with each ribosome fraction was determined by Northern blot analysis using an antisense RNA probe targeted to the 5’ UTR. Northern analysis of transfected cells revealed that under a normal translation condition without treatment, the distribution of HCV IRES-GFP mRNA gradually increased from monosome to polysome, suggesting an increased efficiency of ribosome loading and continued translation. In contrast, IFN-α treatment (IFN+) resulted in an arrest of the majority of HCV IRES-GFP mRNA in the monosome peaks and reduction in the polysome fractions (Figure **5C**, lanes 12-14). Similar results were consistently achieved in three separate experiments. A Similar mechanism is also operative in the case of RBV treatment. Polysome analysis was performed using HCV IRES-GFP transfected cells treated with RBV. The distribution of IRES-GFP mRNA in the RBV treated (RBV+) cells was found in monosome peaks and reduction in polysome peaks (Figure **5D**, lanes 10-14). To address the specificity of IFN-α action on the IRES-GFP mRNA translation, we examined mRNA distribution using EGFP mRNA after IFN-α or RBV treatment. The distribution of GFP mRNA in the polysome fractions was measured by Northern blot analysis using a GFP specific antisense riboprobe. We found no significant difference in the distribution of EGFP mRNA between the monosome and polysome fractions between cells with or without IFN-α (Figure **5E**). To correlate the results of HCV IRES-GFP mRNA distribution profiles in the polysome fractions in the transfected cells with and without IFN treatment, we performed comparative analysis by measuring the density of bands seen in the Northern blot analysis. The band intensity of Northern blots was measured using TatalLab (TL120) software and the values were expressed as a percentage of total RNA recovered in the gradient (Figure **5F**). This analysis clearly shows that both IFN-α and RBV the inhibited loading of polyribosomes to the HCV-IRES containing mRNA. This type of alternation in the mRNA distribution was not observed using control mRNA that is translated via non-IRES mechanism (Figure **5G**).

The article "Interferon and Ribavirin Combination Treatment Synergistically Inhibit HCV Internal Ribosome Entry Site Mediated Translation at the Level of Polyribosome Formation" was retracted in 2024. Reasons: duplicated images; overlap with earlier publications; original data or images not available; unreliable results or conclusions.

**Figure 5:** The distribution of HCV IRES-GFP mRNA in the monosome and polysomes fractions in the Huh-7 cells with (+) and without (-) IFN-α and RBV treatment. (**A**) Illustrates the separation of monosome and polysomes along the sucrose gradient fractions (1 to 14). The values indicate the spectrophotometry of optical density of the polysome fractions at 260 nm wavelengths. The point arrow shows the 60S, 80S and separation between monosomes and polysomes in the gradient fractions. (**B**) Formaldehyde agarose gel electrophoresis and ethidium bromide staining of RNA samples isolated from the corresponding gradient fractions of untreated Huh-7 cells. The 18S and 28S band appears on the gel throughout the fractions and it become more intense on the 80S fractions of the gradient as expected. (**C**) Shows the distribution of HCV IRES-GFP mRNA in the monosome and polysome fractions by Northern blot analysis using a riboprobe targeted to the 5’ UTR. In the untreated IFN (-) cells the IRES-GFP mRNA efficiently translated and formed polyribosome complexes (Lane 11-14). But the IFN treatment (+) prevented polysome formation on IRES-GFP mRNA (Lane 11-14). (**D**) In the RBV untreated Huh-7 cells, the IRES-GFP mRNA efficiently translated and formed polyribosome complexes (Lane 11-14). RBV treatment (+) prevented polysome formation on IRES-GFP mRNA (Lane 10-14). (**E**) Similar experiment was performed where the effect of IFN-α or RBV treatment on the distribution of EGFP mRNA was examined by Northern blotting using RNA probe specific to GFP. IFN-α treatment did not alter the distribution of EGFP mRNA that translates by non-IRES dependent mechanism. (**F**) Comparison of the relative amount of HCV IRES and non-IRES mRNAs in monosome and polysome fractions in the sucrose density gradient analysis generated from the transfected cells. Density of the Northern blot was measured using an image analysis computer software (Total Lab, TL120). Values are expressed as percentage of total mRNA recovered from the gradient versus the mRNA present in each fraction. (**G**) The formation of polyribosome of EGFP mRNA was not altered by IFN-α treatment.

The article "Interferon and Ribavirin Combination Treatment Synergistically Inhibit HCV Internal Ribosome Entry Site Mediated Translation at the Level of Polyribosome Formation" was retracted in 2024. Reasons: duplicated images; overlap with earlier publications; original data or images not available; unreliable results or conclusions.

### RBV treatment altered the association of IMPDH and protein kinase R (PKR) with polysome fractions

To determine whether IMPDH levels could be associated differently in the polysome fractions after RBV treatment which is why inhibited the HCV IRES mediated GFP translation, protein extracts were prepared from monosome and polysome fractions and Western blot analysis was performed. Untreated cells IMPDH, PKR, and pPKR were detectable throughout the gradient (Figure **6A**). IFN-α treatment induced PKR activation and eIF2α phosphorylation. The phosphorylated eIF2α protein was accumulated in the monosome and disome fractions but absent in the polysome fractions (Figure **6B**, lane 6-10). Ribavirin treatment accumulated the IMPDH levels in the monosome and disome fractions but not in the polysome fractions (Figure **6C**). Activated pPKR and peIF2α were also detected in the monosome and disome fractions but not in the polysome fractions (Figure **6C**, lanes 7-10). These results indicated that RBV treatment inhibited distribution of cellular IMPDH, which accumulated in the lower density ribosome fractions.

**Figure 6:** Western blot analysis of polyribosome fractions of HCV IRES-GFP transfected cells. (**A**) Untreated HCV IRES-GFP transfected cells showing IMPDH, PKR, pPKR is bound to the ribosome throughout the gradient. (**B**) PKR induced peIF2α protein is found in the monosome-containing fractions (lanes 1-5) and absent in the higher density polyribosome fractions (lanes 6-10) due to IFN-α treatment. (**C**) IMPDH, pPKR and peIF2α proteins were found in the monosome fractions (lanes 1-6) but excluded from the high-density polyribosome fractions (lanes 6-10). The level of actin was detected throughout the gradient.

### PKR and IMPDH are required for IFN-α and RBV mediated inhibition of HCV IRES-GFP translation

We found the phosphorylation of PKR and eIF2α was increased due to IFN-α or RBV treatment (Figure **7A**). Ribavirin is a synthetic nucleoside analog and known inhibitor of IMPDH enzyme. Ribavirin or IFN-α treatment did not increase or decrease the expression of IMPDH level (Figure **7A**). Inhibition of IMPDH and PKR levels by siRNA restored the inhibitory action of RBV on HCV IRES-GFP translation (Figure **7B and C**). Inhibition of IMPDH activity by RBV is known to decrease the intracellular level of guanosine nucleotide pools resulting in the antiviral activity. Pretreatment with increased concentration of guanoside indeed neutralized the RBV mediated IRES-GFP translation (Figure **7D**). Depletion of the GTP pool caused by the inhibition of IMPDH enzyme activity due to RBV contributes to the inhibition of HCV IRES-GFP translation. We also verified that the inhibition of PKR by siRNA prevented IFN-α mediated inhibition of HCV IRES-GFP translation (Figure **7E and F**). These results suggest that PKR and IMPDH are involved in the IFN-α and RBV mediated synergistic inhibition of HCV IRES mediated translation.

The article "Interferon and Ribavirin Combination Treatment Synergistically Inhibit HCV Internal Ribosome Entry Site Mediated Translation at the Level of Polyribosome Formation" was retracted in 2024. Reasons: duplicated images; overlap with earlier publications; original data or images not available; unreliable results or conclusions.

**Figure 7:** IFN-α and RBV synergy antiviral mechanism involves the activation of PKR, eIF2α and inhibition of cellular IMPDH. (**A**) IFN-α and RBV each induced phosphorylation of PKR and eIF2α. (**B**) Flow cytometric analysis showing RBV show a dose dependent inhibition of HCV IRES-GFP translation. (**C**) Inhibition of IMPDH and PKR levels by siRNA prevented RBV antiviral action against HCV IRES-GFP translation determined by flow cytometric analysis. (**D**) Dose dependent prevention of RBV action due to increasing concentration of guanosine was determined by flow cytometric analysis. (**E**) IFN-α inhibits HCV IRES-GFP translation. (**F**) Inhibition of PKR by siRNA prevented IFN-α mediated inhibition of HCV IRES-GFP translation.

## Discussion

Molecular studies for determining IFN-α antiviral mechansims against HCV are possible due to the availability of highly efficient HCV cell culture systems. Many investigators, including our laboratory, have shown that IFN-α effectively inhibits HCV replication in cell culture model [23,24]. IFN-α binds to the cell surface receptors leading to the activation of Janus kinase signal transducer and activator of transcription (Jak-Stat) pathway. Activation of cellular Jak-Stat pathway results in the phosphorylation and nuclear translocation of the Stat-IRF9 complex to initiate antiviral gene transcription [25]. A number of key antiviral proteins are induced through the activation of the Jak-Stat pathway including the double stranded RNA-activated protein kinase (PKR), 2’5’-oligoadenylate synthethase (2’5’ OAS) and MxA. Studies have shown that IFN-α induced antiviral activity is mediated by interferon inducible ISGs [26]. Mechanisms of IFN-α antiviral activity through the inhibition of HCV IRES mediated translation are supported by a number of studies [27–31]. The newly discovered type III IFN called IFN-λ also inhibits IRES mediated translation of HCV and hepatitis A [32]. There is an agreement that Type I, Type II and Type III IFN inhibit HCV replication by blocking at the level of HCV IRES mediated translation that involves the PKR induced phosphorylation of eIF2α [27,28]. The eIF2α is an eukaryotic initiation factor required for protein translation [33]. This eIF2 protein exists as heterotrimer consisting of eIF-α, eIF-beta and eIF-gamma. The eIF2 protein complexes with GTP and the initiator t-RNA to form the 43S pre-initiation complex. The 43S pre-initiation complex binds to AUG codon on the target mRNA to initiate protein translation. The dissociation of the complex occurs when the eIF2 to hydrolyzes its GTP by eIF5 (a GTPase-activating protein). This conversion causes the eIF-2-GDP to be released from the 48S complex and translation to begin after recruitment of 60S ribosome used and formation of 80S initiation complex. With the help of guanine nucleotide exchange factor eIF2-beta, the eIF2-GDP is exchanged to eIF2-GTP, which initiates another round of translation. The phosphorylation of eIF2α inhibits recycling of this initiation factor and blocks protein synthesis [33].

The article "Interferon and Ribavirin Combination Treatment Synergistically Inhibit HCV Internal Ribosome Entry Site Mediated Translation at the Level of Polyribosome Formation" was retracted in 2024. Reasons: duplicated images; overlap with earlier publications; original data or images not available; unreliable results or conclusions.

The antiviral activity of RBV against HCV is mediated through a number of mechanisms which include: (i) inhibition of cellular IMPDH required for de novo synthesis of guanosine triphosphate, (ii) RBV triphosphate directly inhibits HCV RNA polymerase activity, (iii) RBV can be incorporated into viral genome by HCV RNA polymerase causing mutation in the viral genome, (iv) RBV enhances IFN-α signaling by inducing the expression of interferon-stimulated genes (ISG), (v) RBV also inhibits cellular eIF4E activity required for translation of viral genome, and (vi) RBV helps to clear the virus by stimulating the T helper 1 response of host. Among these candidate mechanisms inhibition of cellular IMPDH by RBV has been verified by a number of laboratories using HCV and other virus infection models [34–37]. Molecular studies of RBV action against HCV are possible due to the availability of *in vitro* cell culture systems. A number of new studies support the RBV antiviral mechanism against HCV replication through inhibition of cellular IMPDH and reduction of GTP pool [37–40]. Mori et al [37] reported that the predominant antiviral mechanism of RBV against HCV is through the inhibition of inosine monophosphate dehydrogenase (IMPDH) not though the error catastrophe, the IFN signaling or oxidative stress. This study is supported by results of other investigators who showed that decrease in GTP also leads to suppression of HCV RNA synthesis by NS5B RNA polymerase [38]. The mechanism of IMPDH inhibition by RBV is supported by the report of Zhou et al [39] indicating that exogenous guanosine suppressed the RBV effect where as potent IMPDH inhibitors MPA and VX-497 enhanced RBV antiviral effect. IMPDH modulates intracellular guanosine nucleotide levels. Therefore it affects a number of cellular processes involved in translation, cell proliferation and RNA/DNA synthesis. IMPDH catalyzes the important step in guanine nucleotide biosynthesis. IMPDH has been shown to be associated with polyribosome, suggesting that this house-keeping gene plays an important role in translational regulation [41]. In our study we found that the distribution of IMPDH is halted in monosome and disome fraction and absent in polysome fractions supporting the role IMPDH in HCV IRES mediated translation.

The article "Interferon and Ribavirin Combination Treatment Synergistically Inhibit HCV Internal Ribosome Entry Site Mediated Translation at the Level of Polyribosome Formation" was retracted in 2024. Reasons: duplicated images; overlap with earlier publications; original data or images not available; unreliable results or conclusions.

Ribavirin in combination with IFN-α showed a marked improvement in the sustained antiviral response in chronic HCV infection. The synergistic antiviral mechanism of IFNα and RBV combination therapy is not known. Only a few studies have been published which explain why RBV and IFN-α combination treatment is highly effective against HCV replication [42–46]. Thomas et al [42] showed that RBV enhanced the IFN-α antiviral activity by inducing the expression of interferon inducible genes (ISGs) and interferon regulatory factor (IRF-7) and (IRF-9). Stevenson et al [43] showed that RBV enhanced IFN-α induced phosphorylation of Stat1, Stat3 and MxA expression and enhanced IFN-α induced cellular Jak-Stat pathway. Liu et al [44] showed that RBV enhances IFN-α signaling through activation of separate antiviral signaling by inducing the expression of cellular p53. This finding is supported by a report indicating that p53 plays an important role in host antiviral defense mechanisms and directly inhibits HCV replication [45]. A previous report by Liu et al [46] indicates that RBV enhances the IFN-α antiviral activity through the up-regulation of PKR activity. None of these studies have shown the synergistic antiviral effect of IFN-α and RBV combination treatment using HCV cell culture. Our results indicate IFN-α and RBV combination treatment synergistically inhibit HCV replication in replicon and infected cell culture models. We show here for the first time that the synergy antiviral action of IFN-α and RBV combination therapy is at the level of inhibition of HCV IRES mediated translation. IFN-α directly inhibits HCV IRES translation by preventing polyribosome loading through PKR mediated eIF2α phosphorylation. Ribavirin inhibits HCV IRES translation by preventing the polyribosome loading of HCV IRES mRNA. Ribavirin mediated blockage of polyribosome loading involves two important mechanisms that involve PKR and IMPDH. Ribavirin mediated PKR and eIF2α phosphorylation inhibits the recycling of eIF2α and inhibits HCV IRES translation. Ribavirin mediated inhibition of IMPDH activity decreases the cellular GTP pool, which inhibits the HCV-IRES translation by preventing polyribosome loading. This is supported by the results showing that pretreatment of guanosine prevented RBV mediated HCV IRES-GFP translation. Based on these observations, we propose a model explaining how RBV mediated depletion of GTP pool and activation of PKR by IFN-α and RBV combination treatment could be playing an important role in the synergy antiviral mechanism (Figure **8**). The detailed mechanism how IFN-α and RBV combination treatment leads to efficient translation arrest of HCV IRES mRNA will be the topic of future investigation.

The article "Interferon and Ribavirin Combination Treatment Synergistically Inhibit HCV Internal Ribosome Entry Site Mediated Translation at the Level of Polyribosome Formation" was retracted in 2024. Reasons: duplicated images; overlap with earlier publications; original data or images not available; unreliable results or conclusions.

**Figure 8:** Diagram summarized the proposed IFN-α and RBV synergy antiviral mechanisms against HCV IRES-GFP translation. IFN-α binds to the cell surface receptor, which activates the cellular Jak-Stat pathway leading to the activation of PKR. The activated PKR phosphorylates the eIF-2α. Phosphorylation of eIF-2α inhibits the recycling of initiation factors and translation initiation. On the other hand, RBV activates the PKR and eIF2 α phosphorylation and inhibits the translation initiation. Ribavirin inhibits HCV IRES translation by inhibiting IMPDH and GTP pool.

## Supporting Information

Figure S1 **HCV genomic and sub-genomic constructs and cell culture models used to study IFN-α and RBV antiviral synergy mechanisms.**
(**A**) HCV full-length JFH1-RLuc chimera clone (13) used in the infectivity assay and sub-genomic HCV RNA used to generate stable S3-GFP replicon cell line (12). (**B**) Structure of pHCV IRES-GFP and pHCV-IRES-Rluc plasmid clone used for this study. The HCV-IRES-sequences were transcribed from T7 promoter and the 3’ UTR sequences were added at the 3’ end of GFP or RLuc. pEGFP-N1 and pDsRed-N1 plasmids were used as controls. (**C**) Shows the steps used to express HCV IRES-GFP or HCV IRES-RLuc using a recombinant adenovirus expressing T7 RNA polymerase.
(TIF)

Figure S2 **MTT assay showing the effect of IFN-α and RBV combination treatment on viability of Huh-7 and S3-GFP cells.**
(**A**) Huh-7 cells were treated with increasing concentration of RBV (10-200 µg/mL) for 48 hours and the viability was measured. (**B**) S3-GFP cells were treated with indicated concentrations of RBV or IFN-α and cell viability was determined at 48 hours. (**C**) Cell viability of combination treatment of IFN-α and RBV at various combinations. S3-GFP cells were treated with different concentration of RBV with one concentration of IFN-α for 48 hours and cell viability was determined by MTT assay.
(TIF)

Figure S3 **Effect of IFN-α and RBV treatment on (A) GFP and (B) Red fluorescence protein (RFP) expression by non-IRES mechanism.**
(TIF)
